The article "Marketplace or Hybrid: Vendor's Information Sharing with e-Retailer" was published in 2022. Journal: Comput Intell Neurosci.

# Marketplace or Hybrid: Vendor's Information Sharing with e-Retailer

**DOI:** 10.1155/2022/7149531

**Published:** 2022-06-28

**Authors:** Dan Li, Kang Li, Xue Pan

**Affiliations:** ^1^School of Business Administration, Shanghai Lixin University of Accounting and Finance, Shanghai 201600, China; ^2^The Research & Development Department, Heilongjiang Ecology Meteorological Centre, Harbin150030, China

## Abstract

This study explores the information sharing (IS) in a supply chain (SC) with a vendor selling goods via an e-retailer to consumers. Four scenarios were considered for the multistage game between the vendor and the e-retailer, and the vendor's policy of IS and the e-retailer's decision on online platform access were discussed under each scenario. The results show that the e-retailer will access the online platform at a low fixed access fee and will not at a high fixed access fee. Whether the vendor shares information with the e-retailer or not, he/she always faces a worse situation with e-retailer's online access. The vendor's decision on IS hinges on the commission rate, contesting intensity, and fixed access fee. When the commission rate is low, the vendor will share the demand if the fixed access fee is low and will not share the information if the access fee is moderate. When the commission rate is high and the contesting is fierce, the vendor is willing to share the demand if the fixed access fee is low or moderate and has no difference in the decision on IS if the fixed access fee is high.

## 1. Introduction

The advance of mobile technology has added momentum to online retailing. Many e-retailers no longer serve as online marketplaces but switch to selling their own-brand goods. The switch triggers the contesting between e-retailers and vendors. Amazon, the leading American e-retailer, has built many own brands, such as Amazon Basics, Presto, and Pinzon. JD.com, a Chinese e-retailer, has joined the online sales contesting and marketed goods of its own brands, namely, Jingzhao and JD Jingxuan.

By opening own-brand stores online, e-retailers could penetrate more related businesses and areas, realize stronger sales growth, and expand their influences. Nevertheless, e-retailers may hesitate to sell their own-brand goods in the lack of demand knowledge. Many large vendors, familiar with good information and understand consumer demand, can collect highly accurate market information. If vendors refuse to share information, e-retailers might not know the potential gains and costs of selling own-brand goods. Hence, the brand expansion policy of e-retailers depends directly on the information sharing (IS) policy of vendors. Based on the information shared by vendors, e-retailers will weigh benefits against costs and might choose to sell own-brand goods. If so, a fierce contesting will ensue between e-retailers and vendors.

The article "Marketplace or Hybrid: Vendor's Information Sharing with e-Retailer" was published in 2022. Journal: Comput Intell Neurosci.

This study considers the IS in a supply chain (SC) with a vendor and an e-retailer. In the SC, the vendor first forecasts the consumer demand and chooses whether to share it with the e-retailer or not. Drawing on the vendor's decision, the e-retailer then chooses to sell own-brand goods through the online platform. Thus, an IS model was introduced with different cases and used to examine the e-retailer's expected gains with and without online access, as well as the impact of several parameters on the expected gains. The relevant results were verified through numerical experiments.

## 2. Literature Review

Our research draws merits from the previous studies on IS in SC and e-retailers' policy of selling modes. Li [1] introduced the IS problem in an SC consisting of several vendors and competitive retailers. Yan et al. [2] analysed how the value of cooperative advertising between retailers and producers impacts IS in a dual platform SC. Shang et al. [3] designed an IS model to reveal the influence of nonlinear production cost, contesting intensity, and contract to charge a payment offered by a retailer over the SC. Dominguez et al. [4] considered partial IS involving retailers with four operating factors and examined the effects of these factors on performance improvement. Some scholars pay attention to bilateral IS problem. Bian et al. [5] investigated the bilateral IS between the producer and retailer in the SC, provided that both sides have the demand knowledge. Wei et al. [6] proposed four decision models under different bilateral IS patterns in two SCs. Zhang and Xiong [7] studied the IS problem in a closed-loop SC with asymmetric demand predictions and developed a model containing two scenarios. Li and Zhang [8] explored the ex-ante IS problem in an SC with a retailer in the downstream and a make-to-stock producer in the upstream. Khan et al. [9] presented an inventory model to quantify the environmental and social costs. Zhang et al. [10] addressed after service deployment and IS policies in an SC with different environments. Wang et al. [11] constructed a Stackelberg game with IS and information concealment scenes and demonstrated the impact of information dissemination.

The emergence of e-retailers has attracted much research attention to e-retailers in the SC and their policy of sales modes. Zhang and Zhang [12] discussed e-retailer's IS decision and vendor's offline platform access policy. Tian et al. [13] investigated the selection between three sales modes and proved that the sharing of market demand between e-retailers mitigates the bullwhip effect on the SC and the vendor's inventory level. Wang et al. [14] put forward four IS models in the online retailing SC with a hybrid format, concluding that platform contesting intensity and proportional transaction fee exert a great effect on the IS policy. Pi and Wang [15] developed game theory models for the dual online platform contesting between an incumbent e-retailer and other e-retailers under different SC structures. Based on the theoretical models, Wei et al. [16] attempted to optimize the online sales formats of e-retailers under the effects of the e-retailers' platform roles, difference in market shares, etc. Guo et al. [17] studied the resales platform structure of online recyclers for waste electrical and electronic equipment (WEEE) and created agency and self-run models to analyse the platform selection of such recyclers. Some scholars extend their research to the competitive strategy between suppliers and retailers. Li et al. [18] presented a game theory model to study the platform and brand policies between a domestic brand producer and a retailer. Zhao et al. [19] evaluated the impact of market demand sharing among e-retailers on the bullwhip effect in the SC and on the inventory level of the only vendor in the SC. Zhang et al. [20] researched the retailer's choice between platform structures and his/her decisions on a good price in an SC with a producer and a retailer. Shi et al. [21] developed a retailer Stackelberg pricing model to evaluate the e-retailers' risk of introducing an additional marketplace platform. Ferreira et al. [22] tried to optimize the pricing decisions of the e-retailer. Chen et al. [23] developed game theory models to explore the promotion decisions, with the aid of the resales and agency sales models, in the presence of fierce contesting between retailers. Assuming that both the vendor and the e-retailer can obtain the demand of online sales, Pei and Yan [24] derived a motivation mechanism for the IS by the vendor and the e-retailer and prevented the information from being distorted. Abhishek et al. [25] introduced a model to explain the e-retailer's selection between the agency sales platform and resales platform. Li et al. [26] focused on IS problem between e-commerce platform with competitive suppliers under different operation modes. The results showed that, in the RR (retail) model, the e-commerce platform has no incentive to share information. However, in the AR (agent + retail) model, the e-commerce platform has no incentive to share information only to suppliers who have opened retail channels. In the AA (agent) model, e-commerce platforms are motivated to share information with two suppliers. Li et al. [27] studied the motivation of retailer to share demand forecasting information with suppliers who have the ability of online sales encroachment. Their findings extended the traditional understanding. The result showed that retailers might share information to encourage suppliers to encroach if the information accuracy of demand forecast or the direct selling cost of suppliers is very low, or if the information accuracy of demand forecast and the direct selling cost of suppliers are both very high. However, retailers tended to keep the information confidential to prevent suppliers from deliberately establishing direct channels.

The article "Marketplace or Hybrid: Vendor's Information Sharing with e-Retailer" was published in 2022. Journal: Comput Intell Neurosci.

The information problem in the SC involving e-retailers is much more complicated than that in a general SC. However, few scholars have paid attention to the IS problem in the SC with competing e-retailers. Zhang and Zhang [12], Tian et al. [13], Wei et al. [16], and Abhishek et al. [25] have considered sales format decisions for e-retailers in different scenarios. Our research has the following differences from their research: (1) unlike Zhang and Zhang [12], Tian et al. [13], and Wei et al. [16], our research studies an SC with a producer selling goods through an e-retailer in an online market mode, rather than an SC with IS problem in traditional wholesale and retail modes [20]; (2) this paper focuses on the vendor's information policy, while they considered the retailer's information policy or two-way information policy; (3) this paper highlights e-retailers' decisions on online platform access, while Abhishek et al. [25] talked about the vendor's decisions on offline access. In these aspects, our study extends the research scope on IS in the SC.

## 3. Model Framework

Our research considers an SC with a vendor (she) selling goods through an e-retailer (he) to consumers. The vendor sets the good price, while the e-retailer makes gains by charging the vendor a commission rate, which is a common practice in the industry. The vendor is assumed to know the demand knowledge better than the e-retailer, thanks to her insights into consumer requirements and experience in consumer service. The e-retailer can choose whether to access an online platform or not, i.e., sell the same goods manufactured by himself. If he chooses to access the online platform, he will not only make gains by charging the commission rate but also benefits from goods directly sold to consumers online. However, the online expansion will bring him a fixed access fee F. If the e-retailer chooses not to access the online platform, the demand function can be given by

(1) $$\begin{array}{c} q=\alpha +\theta -p_{1}, \end{array}$$

where *α* is the deterministic part of potential market demand; *θ* is the demand uncertainty with zero mean and variance *σ*^2^; *p*_1_ and *p*_2_ are the good prices decided by the vendor and the e-retailer, respectively. If the e-retailer accesses the online platform, the demand function can be given by

(2) $$\begin{array}{c} q_{i}=\frac{1}{1-r^{2}}\left(\left(1-r\right)\left(\alpha +\theta \right)-p_{i}+rp_{3-i}\right)\left(i=1,2\right), \end{array}$$

where *q*_1_ and *q*_2_ are the demands of the vendor and the e-retailer, respectively; *r* ∈ (0,1) is the contesting intensity (the greater the *r* value, the more intense the contesting). In operation management, the demand is usually described by a linear function [1, 2].

The article "Marketplace or Hybrid: Vendor's Information Sharing with e-Retailer" was published in 2022. Journal: Comput Intell Neurosci.

The vendor accesses a demand signal Y satisfying *E*[*Y* *|* *θ*]=*θ*, i.e., Y is an unbiased estimator of *θ*. The conditional expectation is linearly correlated with Y. In other words, *E*[*θ* *|* *Y*] can be expressed as follows:

(3) $$\begin{array}{c} E\left[\theta \;|\;Y\right]=\frac{1}{1+t\sigma^{2}}E\left[\theta \right]+\frac{t\sigma^{2}}{1+t\sigma^{2}}Y=\beta \left(t,\sigma \right)Y, \end{array}$$

where *E*[*θ*]=0 and *t*=(1/*E*[*Var*(*Y* *|* *θ*)]) and *β*(*t*, *σ*)=(*tσ*^2^/(1+*tσ*^2^)) are the accuracy and weight of the signal, respectively. According to the common information structure in the relevant literature [3, 4], we have

(4) $$\begin{array}{c} E\left[Y^{2}\right]=Var\left(Y\right)-{\left[E\left(Y\right)\right]}^{2}\\ =Var\left[E\left(Y\;|\;\theta \right)\right]+E\left[Var\left(Y\;|\;\theta \right)\right]\\ =Var\left(\theta \right)+E\left[Var\left(Y\;|\;\theta \right)\right]\\ =\sigma^{2}+\frac{1}{t}. \end{array}$$

Figure 1 shows the timeline of the game of the vendor and the e-retailer in the target SC. At time *t*_1_, the vendor makes the ex-ante decision, whether to share information (S) or not (N) to the e-retailer, before observing the accurate demand, and then accesses the demand knowledge. At time *t*_2_, the e-retailer chooses whether to access the online platform (*E*) or not (F). At time *t*_3_, the vendor sets a good price *p*_1_ and the e-retailer sets a good price *p*_2_, if he accesses the online platform.

In our model, the vendor chooses an IS policy before the e-retailer chooses to access the online platform or not. For the multistage game, our model aims to achieve the subgame-perfect Nash equilibrium. Four cases of the multistage game were considered: SE, SF, NE, and NF. For instance, SE implies that the vendor shares demand knowledge and the e-retailer accesses the online platform. These cases are analysed in detail in the following.

The article "Marketplace or Hybrid: Vendor's Information Sharing with e-Retailer" was published in 2022. Journal: Comput Intell Neurosci.

### 3.1. A-Case SF

In this case, the vendor shares demand knowledge and the e-retailer chooses not to access the online platform. Then, the gains of the vendor and the e-retailer can be expressed as follows:

(5) $$\begin{array}{c} \pi_{s}^{SF}=\left(1-\zeta \right)p_{1}\left(\alpha +E\left[\theta \;|\;Y\right]-p_{1}\right), \end{array}$$

(6) $$\begin{array}{c} \pi_{e}^{SF}=\zeta p_{1}\left(\alpha +E\left[\theta \;|\;Y\right]-p_{1}\right). \end{array}$$

The optimal good price can be derived by maximizing the vendor's gain:

(7) $$\begin{array}{c} p_{1}^{SF}=\frac{\alpha +\beta \left(t,\sigma \right)Y}{2}. \end{array}$$

Substituting the optimal good price into formulas (5) and (6), it is possible to obtain the equilibrium gains for the vendor and the e-retailer:

(8) $$\begin{array}{c} \pi_{s}^{SF*}=\frac{\left(1-\zeta \right){\left(\alpha +\beta \left(t,\sigma \right)Y\right)}^{2}}{4},\\ \pi_{e}^{SF*}=\frac{\zeta {\left(\alpha +\beta \left(t,\sigma \right)Y\right)}^{2}}{4}. \end{array}$$

### 3.2. B-Case SE

In this case, the vendor shares demand knowledge and the e-retailer accesses the online platform. Then, the gains of the vendor and the e-retailer can be expressed as follows:

(9) $$\begin{array}{c} \pi_{s}^{SE}=\left(1-\zeta \right)p_{1}\frac{1}{1-r^{2}}\left(\left(1-r\right)\left(\alpha +E\left[\theta \;|\;Y\right]\right)-p_{1}+rp_{2}\right), \end{array}$$

(10) $$\begin{array}{c} \pi_{e}^{SE}=\zeta p_{1}\frac{1}{1-r^{2}}\left(\left(1-r\right)\left(\alpha +E\left[\theta \;|\;Y\right]\right)-p_{1}+rp_{2}\right) \end{array}$$

where *F* is the fixed access fee for the e-retailer to introduce their own brand products. The optimal good price can be derived by maximizing the vendor's gain and the e-retailer's gain, respectively:

(11) $$\begin{array}{c} p_{1}^{SE}=\frac{\left(1-r\right)\left(2+r\right)\left(\alpha +\beta \left(t,\sigma \right)Y\right)}{4-r^{2}\left(1+\zeta \right)},\\ p_{2}^{SE}=\frac{\left(1-r\right)\left(2+r+r\zeta \right)\left(\alpha +\beta \left(t,\sigma \right)\left.Y\right]\right)}{4-r^{2}\left(1+\zeta \right)}. \end{array}$$

To ensure the positivity of gains and prices, it is assumed that 4 − *r*^2^(1+*ζ*) > 0. Substituting the optimal good price into formulas (9) and (10), it is possible to obtain the equilibrium gains for the vendor and the e-retailer:

(12) $$\begin{array}{c} \pi_{s}^{SE*}=\frac{\left(1-\zeta \right)\left(1-r\right){\left(2+r\right)}^{2}{\left(\alpha +\beta \left(t,\sigma \right)Y\right)}^{2}}{\left(1+r\right){\left(-4+r^{2}\left(1+\zeta \right)\right)}^{2}},\\ \pi_{e}^{SE*}=\frac{\left(1-r\right){\left(\alpha +\beta \left(t,\sigma \right)Y\right)}^{2}\left(\left(1+\zeta \right)\left(4+4r-r^{3}\xi \right)+r^{2}\left(1-\zeta -\zeta^{2}\right)\right)}{\left(1+r\right){\left(-4+r^{2}\left(1+\zeta \right)\right)}^{2}}-F. \end{array}$$

The article "Marketplace or Hybrid: Vendor's Information Sharing with e-Retailer" was published in 2022. Journal: Comput Intell Neurosci.

### 3.3. C-Case NF

In this case, the vendor refuses to share the demand and the e-retailer chooses not to access the online platform. Then, the gains of the vendor and the e-retailer can be expressed as follows:

(13) $$\begin{array}{c} \pi_{s}^{NF}=\left.\left(1-\zeta \right)p_{1}\left(\alpha +E\left[\theta \;|\;Y\right]\right)-p_{1}\right), \end{array}$$

(14) $$\begin{array}{c} \pi_{e}^{NF}=\left.\zeta p_{1}\left(\alpha +E\left[\theta \right]\right)-p_{1}\right). \end{array}$$

The optimal good price can be derived by maximizing the vendor's gain:

(15) $$\begin{array}{c} p_{1}^{NF}=\frac{\alpha +\beta \left(t,\sigma \right)Y}{2}. \end{array}$$

Substituting the optimal good price into formulas (13) and (14), it is possible to obtain the expected gains for the vendor and the e-retailer:

(16) $$\begin{array}{c} E\left(\pi_{s}^{NF*}\right)=\frac{\left(1-\zeta \right)\left(\alpha^{2}+\beta^{2}\left(t,\sigma \right)\left(\sigma^{2}+\left(1/t\right)\right)\right)}{4},\\ E\left(\pi_{e}^{NF*}\right)=\frac{\zeta \left(\alpha^{2}-\beta^{2}\left(t,\sigma \right)\left(\sigma^{2}+\left(1/t\right)\right)\right)}{4}. \end{array}$$

### 3.4. D-Case NE

In this case, the vendor refuses to share the demand and the e-retailer accesses the online platform. Then, the gains of the vendor and the e-retailer can be expressed as follows:

(17) $$\begin{array}{c} \pi_{s}^{NE}=\left(1-\zeta \right)p_{1}\frac{1}{1-r^{2}}\left(\left(1-r\right)\left(\alpha +E\left[\theta \;|\;Y\right]\right)-p_{1}+rp_{2}\right), \end{array}$$

(18) $$\begin{array}{c} \pi_{e}^{NE}=\zeta p_{1}\frac{1}{1-r^{2}}\left(\left(1-r\right)\left(\alpha +E\left[\theta \right]\right)-p_{1}+rp_{2}\right) \end{array}$$

After accessing the online platform, the e-retailer would compete with the vendor in price on the online platform. Because of the first-order condition for optimality, the vendor has an optimal response function $p_{1}=\left(\left(\left(1-r\right)\left(\alpha +\beta \left(t,\sigma \right)Y\right)+r\bar{p_{2}}\right)/2\right)$. For the e-retailer, his optimal response function can be expressed as $p_{2}=\left(\left(\left(1-r\right)\alpha +r\left(1+\zeta \right)E\left(\bar{p_{1}}\right)\right)/2\right)$, where $\bar{p_{1}}$ and $\bar{p_{2}}$ are the conjectured variables of *p*_1_ and *p*_2_, respectively. To get the Nash equilibrium solution, suppose $\bar{p_{i}}=p_{i}$ (*i* = 1,2), that is, the conjectures are consistent with the actual decisions. Then, the optimal good price can be obtained by solving the optimal response functions.

(19) $$\begin{array}{c} p_{1}^{NE}=\left(1-r\right)\left(\frac{\left(2+r\right)\alpha }{4-r^{2}\left(1+\zeta \right)}+\frac{\beta \left(t,\sigma \right)Y}{2}\right), \end{array}$$

(20) $$\begin{array}{c} p_{2}^{NE}=\frac{\left(1-r\right)\alpha \left(2+r+r\zeta \right)}{4-r^{2}\left(1+\zeta \right)}. \end{array}$$

Substituting the optimal good price into formulas (17) and (18), it is possible to obtain the expected gains for the vendor and the e-retailer:

(21) $$\begin{array}{c} E\left(\pi_{s}^{SE*}\right)=\frac{\left(1-\zeta \right)\left(1-r\right)\left(4\alpha^{2}{\left(2+r\right)}^{2}+{\left(-4+r^{2}\left(1+\zeta \right)\right)}^{2}\beta^{2}\left(t,\sigma \right)\left(\sigma^{2}+\left(1/t\right)\right)\right)}{4\left(1+r\right){\left(-4+r^{2}\left(1+\zeta \right)\right)}^{2}}, \end{array}$$

(22) $$\begin{array}{c} E\left(\pi_{e}^{SE*}\right)=\frac{\left(1-r\right)\left(\begin{array}{c} 4\alpha^{2}\left(\left(1+\zeta \right)\left(4+4r-r^{3}\zeta \right)+r^{2}\left(1-\zeta -\zeta^{2}\right)\right)\\ -\zeta {\left(-4+r^{2}\left(1+\zeta \right)\right)}^{2}\beta^{2}\left(t,\sigma \right)\left(\sigma^{2}+\left(1/t\right)\right) \end{array}\right)}{4\left(1+r\right){\left(-4+r^{2}\left(1+\zeta \right)\right)}^{2}}-F. \end{array}$$

**Proposition 1 .**

The article "Marketplace or Hybrid: Vendor's Information Sharing with e-Retailer" was published in 2022. Journal: Comput Intell Neurosci.

Depending on the vendor's IS policy, the e-retailer's best choice on online access is as follows:

- When the vendor shares information, the e-retailer will access the online platform if *F* ≤ *F*_1_ and will not access if *F* > *F*_1_
- When the vendor refuses to share information, the e-retailer will access the online platform if *F* ≤ *F*_2_ and will not access if *F* > *F*_2_

Here, *F*_1_=((*α*^2^+*β*^2^(*t*, *σ*)(*σ*^2^+(1/*t*)))(16 − 16*rζ* − *r*^5^*ζ*(1+*ζ*)^2^+*r*^3^(8*ζ*^2^+8*ζ* − 4)+4*r*^2^(*ζ*^2^ − 3*ζ* − 3)+*r*^4^*ζ*(3+2*ζ* − *ζ*^2^)))/(4(1+*r*)(−4+*r*^2^(1+*ζ*))^2^) and *F*_2_=(2*rζβ*^2^(*t*, *σ*)(*σ*^2^+(1/*t*))(−4+*r*^2^(1+*ζ*))^2^ − *α*^2^(−16+16*rζ*+*r*^5^*ζ*(1+*ζ*)^2^+*r*^3^(−8*ζ*^2^ − 8*ζ*+4) − 4*r*^2^(*ζ*^2^ − 3*ζ* − 3)+*r*^4^*ζ*(−3 − 2*ζ*+*ζ*^2^)))/(4(1+*r*)(−4+*r*^2^(1+*ζ*))^2^).

Proposition 1 implies that once the vendor sets her IS policy, the e-retailer's best choice on online access mainly hinges on the fixed access fee F. Specifically, when the vendor shares demand knowledge, the e-retailer will access the online platform if *F* ≤ *F*_1_. When the vendor refuses to share the demand, the e-retailer will access the online platform if *F* ≤ *F*_2_. Hence, the e-retailer will access the online platform at a small fixed access fee F. Moreover, a relatively accurate signal (a large *t*) pushes up the expected gains of the vendor and the e-retailer, dragging down the access threshold for the e-retailer. In this case, the e-retailer is very likely to access an online platform. This proposition is proved in the Appendix.

The article "Marketplace or Hybrid: Vendor's Information Sharing with e-Retailer" was published in 2022. Journal: Comput Intell Neurosci.

**Proposition 2 .**

Due to product competition with the e-retailer's online access, the vendor is worse off whether she shares information with him or not.

Proposition 2 implies that the vendor always faces a worse situation when the e-retailer accesses the online platform, no matter if she shares information with him or not. In other words, the expected gain of the vendor will decrease after the e-retailer accesses the online platform, whether the information is shared or not. The e-retailer's online access intensifies the contesting, inducing a loss to the vendor. Therefore, the vendor does not want the e-retailer to access the online platform. Furthermore, the vendor faces a growing loss as her contesting with the e-retailer intensifies. This is mainly because intense contesting suppresses the market demand for goods manufactured by the vendor.

According to the e-retailer's decision on online access in Proposition 1, the expected gains of the vendor sharing and not sharing demand knowledge can be, respectively, calculated by

(23) $$\begin{array}{c} E\left(\pi_{s}^{S}\left(F\right)\right)=\left\{\begin{array}{c} \frac{\left(1-r\right)\left(1-\zeta \right){\left(2+r\right)}^{2}f_{1}}{\left(1+r\right){\left(-4+r^{2}\left(1+\zeta \right)\right)}^{2}},\;\text{if }F\leq F_{1},\\ \frac{\left(1-\zeta \right)f_{1}}{4},\;\text{if }F>F_{1}, \end{array}\right. \end{array}$$

(24) $$\begin{array}{c} E\left(\pi_{s}^{N}\left(F\right)\right)=\left\{\begin{array}{c} \frac{\left(1-r\right)\left(1-\zeta \right)f_{2}}{4\left(1+r\right){\left(-4+r^{2}\left(1+\zeta \right)\right)}^{2}},\;\text{if }F\leq F_{2},\\ \frac{\left(1-\zeta \right)f_{1}}{4},\;\text{if }F>F_{2}, \end{array}\right. \end{array}$$

where *E*(*π*_*s*_^*S*^(*F*)) is the expected gain of the vendor when she shares demand knowledge. *f*_1_=(*α*^2^+*β*^2^(*t*, *σ*)(*σ*^2^+(1/*t*))) and *f*_2_=4*α*^2^(2+*r*)^2^+(−4+*r*^2^(1+*ζ*))^2^*β*^2^(*t*, *σ*)(*σ*^2^+(1/*t*)).

**Proposition 3 .**

When the commission rate 0 < *ξ* ≤ *ξ*_1_, the vendor will make the following decisions on whether to share the demand:

- *E*(*π*_*s*_^*S*^(*F*)) > *E*(*π*_*s*_^*N*^(*F*)): if *F* *≤* *F*_*2*_, the vendor will share the demand
- *E*(*π*_*s*_^*S*^(*F*)) < *E*(*π*_*s*_^*N*^(*F*)): if *F*_*2*_*<F* *≤* *F*_*1*_, the vendor will not share the demand
- *E*(*π*_*s*_^*S*^(*F*))=*E*(*π*_*s*_^*N*^(*F*)): if *F* *>* *F*_*1*_, the vendor will be neutral about the IS with the e-retailer

The scenarios of *ζ*_1_ ∈ (0,1) are given in the Appendix.

Proposition 3 implies that, at a low commission rate, the vendor is willing to share the demand if the fixed access fee is low, does not wish to share the information if the said cost is moderate, and remains neutral about IS if the said cost is high. Specifically, when the commission rate and the fixed access fee are both low, the e-retailer always chooses to access the online platform. Then, the best choice of the vendor is to share the demand, which will benefit her. When the commission rate is low and the fixed access fee is moderate, the e-retailer is uncertain about whether to access the online platform. As shown in Proposition 2, the vendor is worse off with e-retailer's online access and would therefore prevent the e-retailer from accessing the online platform. For this purpose, the vendor will not share the demand, such as to increase the access threshold for the e-retailer and prevent the e-retailer from selling the same goods on the online platform. When the commission rate is low and the fixed access fee is high, the e-retailer will not access the online platform. In this case, the expected gain of the vendor is independent of the sharing of demand knowledge.

The article "Marketplace or Hybrid: Vendor's Information Sharing with e-Retailer" was published in 2022. Journal: Comput Intell Neurosci.

**Proposition 4 .**

When the commission rate *ξ*>*ξ*1 and the contesting intensity r> r1, the vendor will make the following decisions on whether to share the demand:

- *E*(*π*_*s*_^*S*^(*F*)) > *E*(*π*_*s*_^*N*^(*F*)): if *F* ≤ *F*_2_, the vendor will share the demand
- *E*(*π*_*s*_^*S*^(*F*))=*E*(*π*_*s*_^*N*^(*F*)): if *F* > *F*_1_, there is no difference for the vendor's decision on IS

The scenarios of *r*_1_ ∈ (0,1) are provided in the Appendix.

Proposition 4 implies that when the commission rate is high and the contesting is fierce, the vendor is willing to share the demand if the fixed access fee is low or moderate and there is no difference for the vendor's decision on IS if the said cost is high. Intuitively, the e-retailer faces a low access threshold facing a high commission rate and a fierce contesting. Hence, he will willingly access the online platform if the fixed access fee is low or moderate. Moreover, if the fixed access fee is low, the e-retailer will access the online platform and the best choice of the vendor is to share the demand. If the fixed access fee is moderate, *F*_1_<*F*_2_, the access threshold will be lowered for the e-retailer, that is, the e-retailer is more willing to access the online platform if the vendor refuses to share information. To prevent the e-retailer from selling the same goods on the online platform, the vendor will decide to share the demand and inform the e-retailer about the exact market potential. Similarly, when the commission rate is high and the contesting is fierce, the e-retailer will not access the online platform at a low fixed access fee. In this case, the expected gain of the vendor will remain the same, irrespective of the sharing or withholding of the demand knowledge.

The article "Marketplace or Hybrid: Vendor's Information Sharing with e-Retailer" was published in 2022. Journal: Comput Intell Neurosci.

## 4. Numerical Examples

Numerical experiments were performed to test the above propositions. The expected gains of the vendor and e-retailer were examined in detail. Referring to Shang et al. [3]'s work, the parameters were configured as follows: *α* = 4, *σ*2 = 1, *ζ* = 0.2, *r* = 0.5, and *t* = 0.9.

If the supplier decides to share information, as shown in Figure 2, if *F* ≤ *F*_1_ (*F*_1_ = 2.865), the e-retailer's expected gain with online access is higher than that without online access, when the vendor shares demand knowledge. If *F* ≤ *F*_2_ (*F*_2_ = 2.273), the e-retailer's expected gain with online access is larger than that without online access, when the vendor refuses to share the demand. Furthermore, if *F* > *F*_1_ (*F*_1_ = 2.865), the e-retailer's expected gain without online access is greater than that with online access, when the vendor shares demand knowledge. If *F* > *F*_2_ (*F*_2_ = 2.273), the e-retailer's expected gain without online access is above that with online access, when the vendor refuses to share the demand. Consequently, whether the vendor chooses to share demand knowledge or not, the e-retailer is willing to access the online platform at a small fixed access fee F and refuses to do so at a large F. If the fixed access fee F is moderate, the e-retailer's decision on online access hinges on the vendor's policy of demand IS. In other words, when the fixed access fee F is moderate, the e-retailer accesses the online platform if the vendor shares demand knowledge, whereas the e-retailer chooses not to access the online platform, if the vendor refuses to share the demand.

To disclose its impact on the expected gain of the vendor, the commission rate *ξ* was adjusted from 0 to 0.9 and the variation in the expected gain was calculated. As shown in Figure 3, with the increase of *ξ*, the expected gain of the vendor decreases, whether the e-retailer accesses the online platform or not. That is, the growing commission rate paid by the vendor will increase the cost, causing a loss to her expected gain.

The vendor's expected gain with IS is larger than that in the absence of IS, when the e-retailer accesses the online platform. Moreover, the vendor's expected gain without e-retailer's online access is greater than that with e-retailer's online access. Thus, the vendor is worse off with e-retailer's online access, whether she shares information to the e-retailer or not.

Figure 4 shows the impact of contesting intensity *r* on the vendor's expected gain. It can be inferred that, with the increase in *r*, the vendor's expected gain decreases, when the e-retailer accesses the online platform. That is to say, the e-retailer's decision of accessing the online platform causes the production contesting between him and the vendor, which will suppress the vendor's expected gain. The contesting intensity *r* has no influence on the vendor's expected gain, when the e-retailer chooses not to access the online platform.

The article "Marketplace or Hybrid: Vendor's Information Sharing with e-Retailer" was published in 2022. Journal: Comput Intell Neurosci.

Furthermore, the vendor's expected gain falls more slowly with the increase in *r*, when the vendor shares information, and the e-retailer accesses the online platform. The main reason is that demand IS with the e-retailer enables her to set a more effective price, which will bring her more benefits.

Figure 5 displays the impact of F on the expected gain of the vendor at different commission rates F. As shown in Figure 5(a), at a low commission rate *ξ* = 0.2, the vendor will share the demand if *F* ≤ 2.273 and will not share the information if 2.273 ≤ *F* ≤ 2.865. The vendor has preference for IS or not if *F* > 2.865. As shown in Figure 5(b), when the commission rate is high (*ξ* = 0.9), the vendor is willing to share the demand if *F* ≤ 2.051 and her expected gain remains the same if *F* > 2.051. A high commission rate *ξ* often leads to a large *F*_2_, i.e., a low access threshold for the e-retailer. Hence, the vendor is willing to share the demand with the e-retailer, giving him more accurate market information. Then, the e-retailer may not access the online platform, especially when the access fee is not very low. The no access scenario will significantly benefit the vendor.

## 5. Conclusions

This study deals with the novel problem of IS in an SC with a vendor selling goods through an e-retailer to consumers. In the problem, the vendor decides whether to share the demand and the e-retailer chooses whether to access the online platform. It was expected that based on the vendor's policy of IS, the e-retailer will access the online platform at a low access fee and will not at a high access fee. The vendor always faces a worse situation with the e-retailer's online access whether she shares information to the e-retailer or not. Moreover, if the commission rate is low, the vendor will share the demand at a low fixed access fee and will not do so at a moderate fixed access fee. When the commission rate is high and the contesting is fierce, the vendor will share the demand if the fixed access fee is low or moderate. There is no difference for the vendor's decision on sharing information, facing a high fixed access fee.

Through numerical analysis, the authors examined the e-retailer's expected gains with and without online access, as well as the influence of parameters such as *ξ*, *r*, and F over the vendor's expected gain. It was observed that whether the vendor shares demand knowledge, the e-retailer is willing to access the online platform at a small fixed access fee F and refuses to do so at a high F value. If the fixed access fee F is moderate, the e-retailer's decision on online access hinges on the vendor's policy of demand IS. Furthermore, with the increase in *ξ* and *r*, the vendor's expected gains with and without e-retailer's online access decreases, when the e-retailer chooses to access the online platform. When the fixed access fee is moderate, the vendor will not share the demand if the commission rate is low and will share the demand if the commission rate is high.

The article "Marketplace or Hybrid: Vendor's Information Sharing with e-Retailer" was published in 2022. Journal: Comput Intell Neurosci.

This research will be further extended to SCs with competitive vendors, resulting in novel SC structures and interesting conclusions. Since the e-retailer can collect and process online demand knowledge, future research will consider the two-way IS between the vendor and the e-retailer.

## Figures and Tables

**Figure 1:** Timeline.

**Figure 2:** Expected gains of e-retailer accessing and not accessing online platform.

**Figure 3:** Impacts of *ξ* on the expected gains of vendor.

**Figure 4:** Impacts of *r* on the expected gains of vendor.

**Figure 5:** Impacts of F on the expected gains of vendor. (a) *ξ* = 0.2. (b) *ξ* = 0.9.

## Data Availability

The data used to support the findings of this study are available from the corresponding author upon request.

## Appendix

Proof of Proposition 1. If the vendor shares information, we have

(A.1) $$\begin{array}{c} E\left(\pi_{e}^{SE*}\right)-E\left(\pi_{e}^{SF*}\right)=\frac{\left(\alpha^{2}+\beta^{2}\left(t,\sigma \right)\left(\sigma^{2}+\left(1/t\right)\right)\right)M_{1}}{4\left(1+r\right){\left(-4+r^{2}\left(1+\zeta \right)\right)}^{2}}-F, \end{array}$$

where *M*_1_=(16 − 16*rζ* − *r*^5^*ζ*(1+*ζ*)^2^+*r*^3^(8*ζ*^2^+8*ζ* − 4)+4*r*^2^(*ζ*^2^ − 3*ζ* − 3)+*ζr*^4^(−*ζ*^2^+2*ζ*+3)). Note that *E*(*π*_*e*_^*SE∗*^) − *E*(*π*_*e*_^*SF∗*^) ≥ 0 if *F* ≤ *F*_1_ and *E*(*π*_*e*_^*SE∗*^) − *E*(*π*_*e*_^*SF∗*^) < 0 if *F* > *F*_1_. When the vendor refuses to share information, we have

(A.2) $$\begin{array}{c} E\left(\pi_{e}^{NE*}\right)-E\left(\pi_{e}^{NF*}\right)=\frac{2r\zeta {\left(-4+r^{2}\left(1+\zeta \right)\right)}^{2}\beta^{2}\left(t,\sigma \right)\left(\sigma^{2}+\left(1/t\right)\right)+\alpha^{2}M_{1}}{4\left(1+r\right){\left(-4+r^{2}\left(1+\zeta \right)\right)}^{2}}-F. \end{array}$$

Note that *E*(*π*_*e*_^*NE∗*^) − *E*(*π*_*e*_^*NF∗*^) ≥ 0 if *F* ≤ *F*_2_ and *E*(*π*_*e*_^*NE∗*^) − *E*(*π*_*e*_^*NF∗*^) < 0 if *F* > *F*_2_.

The article "Marketplace or Hybrid: Vendor's Information Sharing with e-Retailer" was published in 2022. Journal: Comput Intell Neurosci.

Proof of Proposition 2. When the vendor shares information, we have

(A.3) $$\begin{array}{c} E\left(\pi_{s}^{SE*}\right)-E\left(\pi_{s}^{SF*}\right)=\frac{r\left(\alpha^{2}+\beta^{2}\left(t,\sigma \right)\left(\sigma^{2}+\left(1/t\right)\right)\right)\left(-1+\zeta \right)M_{2}}{4\left(1+r\right){\left(-4+r^{2}\left(1+\zeta \right)\right)}^{2}}<0,\\ E\left(\pi_{s}^{NE*}\right)-E\left(\pi_{s}^{NF*}\right)=\frac{r\left(-1+\zeta \right)\left(2\beta^{2}\left(t,\sigma \right)\left(\sigma^{2}+\left(1/t\right)\right){\left(-4+r^{2}\left(1+\zeta \right)\right)}^{2}+\alpha^{2}M_{3}\right)}{4\left(1+r\right){\left(-4+r^{2}\left(1+\zeta \right)\right)}^{2}}<0, \end{array}$$

where *M*_2_=16+*r*(4 − 8*ζ*+*r*(−4 − 8*ζ*+*r*(1+*r*)(1+*ζ*)^2^)) and *M*_3_=16+*r*(4 − 8*ζ*)+*r*^3^(1+*ζ*)^2^+*r*^4^(1+*ζ*)^2^ − 4*r*^2^(1+2*ζ*). It can be easily obtained that *M*_3_^″^(*ζ*)=2*r*^3^(1+*r*) > 0, which implies that *M*_3_(*ζ*) is convex in *ζ*. Note that *M*_3_′(*ζ*)=*r*(−8+*r*(−8+2*r*(1+*r*)(1+*ζ*))) < 0, *M*_3_(0)=16+*r*(1+*r*)(*r*^2^ − 4) > 0, and *M*_3_(1)=16+*r*(−4 − 12*r*+4*r*(1+*r*)) > 0. Hence, *M*_3_(*ζ*) > 0 holds for all *ζ* ∈(0,1). Thus, we have *E*(*π*_*s*_^*SE∗*^) − *E*(*π*_*s*_^*SF∗*^) < 0. Similarly, it can be easily obtained that *E*(*π*_*s*_^*SE∗*^) − *E*(*π*_*s*_^*SF∗*^) < 0.

Proof of Proposition 3. Note that

(A.4) $$\begin{array}{c} F_{1}-F_{2}=\frac{-\beta^{2}\left(t,\sigma \right)\left(\sigma^{2}+\left(1/t\right)\right)g\left(\zeta \right)}{4\left(1+r\right){\left(-4+r^{2}\left(1+\zeta \right)\right)}^{2}}<0, \end{array}$$

where *g*(*ζ*)=−16+48*rζ*+3*r*^5^*ζ*(1+*ζ*)^2^ − 4*r*^2^(−3 − 3*ζ*+*ζ*^2^)+*r*^4^*ζ*(−3 − 2*ζ*+*ζ*^2^) − 4*r*^3^(−1+6*ζ*+6*ζ*^2^). We have *g*′(*ζ*)=*r*(48+*r*(12 − 8*ζ*) − 24*r*^2^(1+2*ζ*)+*r*^3^(−3 − 4*ζ*+3*ζ*^2^)+3*r*^4^(1+4*ζ*+3*ζ*^2^)) and *g*^″^(*ζ*)=−8*r*^2^ − 48*r*^3^+2*r*^4^*ζ*+6*r*^5^*ζ*+12*r*^5^(1+*ζ*)+2*r*^4^(−2+2*ζ*). Define *f*(*ζ*)=*g*^″^(*ζ*); we derive that *f*′(*ζ*)=6*r*^4^+18*r*^5^ > 0. Thus, *f*(*ζ*) increases with *ζ*. Since *f*(0)=4*r*^2^(3*r*^3^ − *r*^2^ − 12*r* − 2) < 0 and *f*(1)=2*r*^2^(15*r*^3^+*r*^2^ − 24*r* − 4) < 0, we can derive that *f*(*ζ*) < 0 for all *ζ*∈(0,1). Then, *g*^″^(*ζ*) < 0. Note that *g*′(0)=*r*(3*r*^4^ − 3*r*^3^ − 12*r*^2^+12*r*+48) > 0 and *g*′(1)=*r*(24*r*^4^ − 4*r*^3^ − 72*r*^2^+4*r*+48) > 0; it can be easily obtained that *g*′(*ζ*) > 0 for all *ζ*∈(0,1). We have *g*(0)=−16+12*r*^2^+4*r*^3^ ≤ 0 and *g*(1)=−16+48*r*+12*r*^5^+20*r*^2^ − 4*r*^4^ − 44*r*^3^. Define *k*(*r*)=*g*(1)=−16+48*r*+12*r*^5^+20*r*^2^ − 4*r*^4^ − 44*r*^3^; we can derive that *k*′(*r*)=48+60*r*^4^+40*r* − 16*r*^3^ − 132*r*^2^ ≥ 0. Since *k*(0)=−16 < 0 and *k*(1)=16 > 0, there exists a unique threshold value *r*_1_ satisfying *k*(*r*_*1*_) *=* *0* such that *k(r)* *>* *0* if *r* *>* *r*_*1*_ and k(*r*) ≤0 otherwise. When *r* ≤ *r*_1_, we can obtain that *g*(0) ≤ 0, *g*(1) ≤ 0, *g*(*ζ*) ≤ 0, and *F*_1_ ≥ *F*_2_. When *r* *>* *r*_*1*_, *g*(0) ≤ 0 and *g*(1) > 0, and there exists a unique threshold value *ζ*_1_ satisfying *g*(*ζ*_1_)=0 such that *g*(*ζ*) ≤ 0 if 0 < *ζ* ≤ *ζ*_1_ and *g*(*ζ*) > 0 if *ζ* > *ζ*_1_. Therefore, it can be easily obtained that *F*_1_ ≥ *F*_2_ if *r* *>* *r*_*1*_ and 0 < *ζ* ≤ *ζ*_1_, whereas *F*_1_ < *F*_2_ if *r* *>* *r*_*1*_ and *ζ* > *ζ*_1_. If *r* ≤ *r*_1_, when *F* ≤ *F*_2_, we have

(A.5) $$\begin{array}{c} E\left(\pi_{s}^{S}\left(F\right)\right)-E\left(\pi_{s}^{N}\left(F\right)\right)=\frac{\left(1-r\right)r\left(-1+\zeta \right)\beta^{2}\left(t,\sigma \right)\left(\sigma^{2}+\left(1/t\right)\right)M_{4}}{4\left(1+r\right){\left(-4+r^{2}\left(1+\zeta \right)\right)}^{2}}>0, \end{array}$$

where *M*_4_=−16+*r*^3^(1+*ζ*)^2^ − 4*r*(3+2*ζ*). If *r* ≤ *r*_1_, when *F*_2_ < *F* ≤ *F*_1_, we have

(A.6) $$\begin{array}{c} E\left(\pi_{s}^{S}\left(F\right)\right)-E\left(\pi_{s}^{N}\left(F\right)\right)=\frac{r\left(\alpha^{2}+\beta^{2}\left(t,\sigma \right)\left(\sigma^{2}+\left(1/t\right)\right)\right)M_{5}}{4\left(1+r\right){\left(-4+r^{2}\left(1+\zeta \right)\right)}^{2}}<0, \end{array}$$

where *M*_5_=16(−1+*ζ*)+*r*^3^(−1+*ζ*)(1+*ζ*)^2^+*r*^4^(−1+*ζ*)(1+*ζ*)^2^+*r*^2^(4+4*ζ* − 8*ζ*^2^) − 4*r*(1 − 3*ζ*+2*ζ*^2^). If *r* ≤ *r*_1_, when *F* > *F*_1_, we have

(A.7) $$\begin{array}{c} E\left(\pi_{s}^{S}\left(F\right)\right)-E\left(\pi_{s}^{N}\left(F\right)\right)=0. \end{array}$$

There is no difference for the vendor in sharing information decisions. If *r* > *r*_1_ and 0 < *ζ* ≤ *ζ*_1_, the expected gains of the vendor are the same.

The article "Marketplace or Hybrid: Vendor's Information Sharing with e-Retailer" was published in 2022. Journal: Comput Intell Neurosci.

Proof of Proposition 4. If *r* > *r*_1_ and *ζ* > *ζ*_1_, when *F* ≤ *F*_1_, we have

(A.8) $$\begin{array}{c} E\left(\pi_{s}^{S}\left(F\right)\right)-E\left(\pi_{s}^{N}\left(F\right)\right)=\frac{\left(1-r\right)r\left(-1+\zeta \right)\beta^{2}\left(t,\sigma \right)\left(\sigma^{2}+\left(1/t\right)\right)M_{4}}{4\left(1+r\right){\left(-4+r^{2}\left(1+\zeta \right)\right)}^{2}}>0. \end{array}$$

If *r* > *r*_1_ and *ζ* > *ζ*_1_, when *F*_1_ < *F* ≤ *F*_2_, we have

(A.9) $$\begin{array}{c} E\left(\pi_{s}^{S}\left(F\right)\right)-E\left(\pi_{s}^{N}\left(F\right)\right)=\frac{r\left(1-\zeta \right)M_{6}}{4\left(1+r\right){\left(-4+r^{2}\left(1+\zeta \right)\right)}^{2}}>0, \end{array}$$

where *M*_6_=2*β*^2^(*t*, *σ*)(*σ*^2^+(1/*t*))(−4+*r*^2^(1+*ζ*))^2^+*α*^2^(16+*r*(4 − 8*ζ*)+*r*^3^(1+*ζ*)^2^+*r*^4^(1+*ζ*)^2^ − 4*r*^2^(1+2*ζ*)). If *r* > *r*_1_ and *ζ* > *ζ*_1_, when *F* > *F*_2_, we have

(A10) $$\begin{array}{c} E\left(\pi_{s}^{S}\left(F\right)\right)-E\left(\pi_{s}^{N}\left(F\right)\right)=0. \end{array}$$

Hence, there is no difference for the vendor in sharing information decisions.
